The article "Application of Quality Control Circle in Promoting the Use of Rubber Dams in the Root Canal Treatment of Primary Teeth" was retracted in 2024. Reasons: suspected computer-generated content; unreliable results or conclusions; concerns about the data; concerns about the results or conclusions.

# Application of Quality Control Circle in Promoting the Use of Rubber Dams in the Root Canal Treatment of Primary Teeth

**DOI:** 10.1155/2020/5397838

**Published:** 2020-02-24

**Authors:** Fang Jingxian, Liu Yang, Liu Qiong, Qian Hong, Liu Hedi, Zhang Jinglan, Liu Fang, Yang Jing, Wu Xiaoming, Song Yingying

**Affiliations:** Department of Pediatric Dentistry, Stomatological Hospital, Southern Medical University, Guangzhou 510280, China

## Abstract

**Objective:**

Study the effect of quality control circle (QCC) in promoting the usage of rubber dams (RD) in root canal treatment of chronic pulpitis in primary teeth.

**Methods:**

Set up a quality control group to increase the amount of rubber dams used in the treatment of chronic pulpitis in primary teeth. Monthly monitoring results of the usage amount were counted by the outpatient computer system. Relevant data were collected through questionnaires, and causes of low utilization were analyzed, and the improvement measurements were formulated and implemented. Quality control circle activity was evaluated.

**Results:**

Through the quality control circle activity, the consumption of rubber dams in the root canal treatment of chronic pulpitis was significantly improved, children in treatment became more cooperative, and operation time of root canal treatment has also been shortened.

**Conclusion:**

The quality control circle activities played a significant role in promoting the use of rubber dams in the root canal treatment of primary teeth, and it can be used as a method to promote new clinical treatment programs.

## 1. Introduction

There are many advantages of using rubber dam (RD) in root canal treatment of chronic pulpitis of deciduous teeth [1], such as improving infection control quality, safety, and therapeutic effects [2, 3]. Therefore, it should be vigorously promoted and applied. However, the utilization rate of rubber dam in deciduous teeth in China is not high in clinical practice [4]. Quality control circle (QCC) is a group of workers who do the same or similar work, who meet regularly to identify, analyze, and solve work-related problems [5]. They are problem solving teams which use simple statistical methods to research and decide on solutions to workshop problems [6]. And they follow the “PDCA” (plan-do-check-act) process [7]. In order to find out the reason why usage of rubber dam was so low in the treatment of chronic pulpitis and to further solve the problem, the following work has been carried out. It has been monitored the usage of rubber dam in root canal treatment of chronic pulpitis of deciduous teeth in the Department of Pediatric Dentistry, Stomatological Hospital of Southern Medical University for twelve months. Through applying quality control circle, the consumption and using techniques of rubber dam has been improved when compared with the previous year. And the quality control circle activity can be used as a method to promote new clinical treatment programs. The details are reported below.

The article "Application of Quality Control Circle in Promoting the Use of Rubber Dams in the Root Canal Treatment of Primary Teeth" was retracted in 2024. Reasons: suspected computer-generated content; unreliable results or conclusions; concerns about the data; concerns about the results or conclusions.

## 2. Materials and Methods

### 2.1. General Information

Our department is the outpatient of Pediatric Dentistry Department in the Tertiary Stomatological Hospital. There are 9 pedodontists, 20 nurses, and 8 dental residents during the year of 2018.

### 2.2. Methods

#### 2.2.1. QCC

Set up a quality control circle group which consists of 11 members, including 10 dentists and 1 nurse.

#### 2.2.2. Topic Selection

The theme of QCC activity is to increase the usage of rubber dam in root canal treatment of chronic pulpitis of deciduous teeth. The event was held from January 2018 to December 2018.

#### 2.2.3. Reason Analysis

Through literature review, brainstorming, and questionnaire, the QCC team analyzed the main reasons for low usage of rubber dam in the treatment of chronic pulpitis of milk teeth as several aspects, and finally determined the improvement measurement as scheduled and improves the operation.

#### 2.2.4. Setting Target

Value of the goal setting formula = current situation value + (improvement value × improvement focus × circle capacity), the amount of rubber dam used before improvement was 20 pieces/(month · dental chair), the circle capacity was assessed and calculated by all circle members as 83.08%, and the target value after improvement was 34 pieces/(month · dental chair), with an improvement range of 66.46%.

#### 2.2.5. Countermeasures Formulation and Implementation

1. Videos about advantages and disadvantages of using rubber dams were played in the waiting room; operating procedures were shown as well
2. Using children's language
3. Normalizing the practice. The rubber dam was placed by means of wing method. According to the tooth position, the rubber dam was drilled, fixed on the rubber dam clamp, and then extended with the rubber dam clamp, and then placed on the tooth neck together with the rubber cloth. During the process, attention was paid to the protection of oral soft tissue, and fingers were used to guide the rubber dam into position [8]
4. Internal and external experience exchanges. Experiences were shared among dentists to face those special tooth conditions
5. Local anesthesia
6. Questionnaire. Survey was conducted to confirm, review, and improve the implementation status and effect
7. Data analysis. Theme progress of rubber dams at each dental chair was counted, and the children in rubber dam group (experimental group) and without rubber dam group (control group) were scored according to Houpt's evaluation scale (Table 1) [9], and the chairside operation time as well as the complications before and after treatment were analyzed

The article "Application of Quality Control Circle in Promoting the Use of Rubber Dams in the Root Canal Treatment of Primary Teeth" was retracted in 2024. Reasons: suspected computer-generated content; unreliable results or conclusions; concerns about the data; concerns about the results or conclusions.

### 2.3. Statistical Analyses SPSS20.0 Software Was Used for Statistical Analysis

The whole process score of Houpt's score and the operation time beside the chair were compared by *t* test, the monthly amount of rubber dam, and the numbers of intraoperative and postoperative complications were compared by chi-square test, and *P* < 0.05 was considered statistically significant.

## 3. Results

### 3.1. Monthly Consumption of Rubber Dam for Milk Teeth in Root Canal Treatment of Chronic Pulpitis Is Promoted by QCC Activities

The activity of quality control circle increased the use of rubber dam in root canal treatment of chronic pulpitis of deciduous teeth in our department. After improvement, consumption of rubber dam was 91pieces per month. Target rate = (improved‐base)/(target‐present) × 100% = (91‐20)/(34‐20) × 100% = 507.14%. Meanwhile, when we compare the patient's amount each month, data shows a similar trend while compared with the year of 2017.

### 3.2. Using Rubber Dam Can Improve the Cooperation Degree and Reduce the Operation Time beside the Chair

The Houpt scores of children in both the experimental group and the control group during the whole process of treatment were assessed, and the chairside operation time were counted too (Table 2). Those results were statistically analyzed, and the difference was statistically significant (*P* < 0.05). The children in the experimental group had a higher degree of cooperation in the treatment, and the use of rubber dam shortened the total treatment time.

### 3.3. Complications of Using Rubber Dam

Intraoperative and postoperative complications of the root canal treatment in both the experimental group and the control group were evaluated by questionnaires and statistical analysis. There were statistical differences on discomfort and gingival bleeding between two groups and mucosal bleeding caused by intraoperative saliva suction could be found in the control group, suggesting that painless anesthesia and pain control techniques should be further improved before root canal treatment (Table 3).

## 4. Discussion

Rubber dam for milk teeth was introduced into our department to use since 2017, but usage amount and frequency was much lower than that for permanent teeth. Based on the fact that the clinical pathway of hospital information management has been included in the treatment of chronic pulpitis of deciduous teeth, the theme of QCC activity is to increase the usage of rubber dam in root canal treatment of chronic pulpitis of deciduous teeth.

The article "Application of Quality Control Circle in Promoting the Use of Rubber Dams in the Root Canal Treatment of Primary Teeth" was retracted in 2024. Reasons: suspected computer-generated content; unreliable results or conclusions; concerns about the data; concerns about the results or conclusions.

Rubber dam in root canal treatment has been recognized as a standard treatment procedure internationally [10]. In developed countries, rubber dams have been widely used in children's oral treatment. A questionnaire survey study among dentists from China and Japan [11] analyzed the application of rubber dam in the treatment of pulp disease of deciduous teeth. The comparative analysis showed that 81.3% of dentists in the Japanese group routinely used rubber dam in the treatment of pulp disease of deciduous teeth, while 38.1% of dentists in the Chinese group used rubber dam, which was significantly lower than that in the Japanese group. Pediatric dentistry in China started late as an independent specialty, with uneven development in different regions. Meanwhile, China has a large population and insufficient resources in specialized hospitals. Dentists in general hospitals also undertake a large number of children's dental diagnosis and treatment. Statistics show that [4] the utilization rate of rubber dam in the affiliated dental hospital is significantly higher compared with the dental department of the tertiary general hospital. In the tertiary general hospital, the use of rubber dam was not popular. Applying dental dam in deciduous teeth root canal therapy has unique advantages [2, 3]. First, children have more saliva and small mouth angle. Compared with the conventional cotton isolation, application of dental dam leads operating space to be relatively clean and dry. It also reduces chances of infection, so as to improve the quality and efficiency of the root canal treatment [12]. Second, the oral mucosa of children is more vulnerable to be impaired than that of adults. Rubber dams can reduce the stimulation and injury of oral soft tissues caused by the dental instruments and medications during root canal treatment. However, there are many reasons for the low utilization rate of rubber dam in the treatment of milk teeth in China [13]. Old dentists were unfamiliar with the rubber dam system and children were afraid of needle injection or rubber dam clamping [14]. In the process of root canal treatment of deciduous teeth without rubber dam, selection of lotion and treatment will be affected to certain extent. Moreover, children with low degree of coordination are likely to swallow or inhale dental instrument materials [15], which will cause unnecessary medical disputes. In Table 3, it has been shown that rubber clamp itself may cause intraoperative discomfort and bleeding during operation. The suitability between the crown and the rubber dam of the baby teeth still needs further improvement. Therefore, the use of milk teeth rubber dam requires the joint efforts of child, parents, dentists, and nurses [16]. In addition to communication and technical training for both dentists and nurses, the advantages and values of using rubber dams must be emphasized and routine usage should be encouraged. Besides, more suitable rubber dam clamp for Chinese children should be developed.

The article "Application of Quality Control Circle in Promoting the Use of Rubber Dams in the Root Canal Treatment of Primary Teeth" was retracted in 2024. Reasons: suspected computer-generated content; unreliable results or conclusions; concerns about the data; concerns about the results or conclusions.

In order to improve the application, several methods have been used, such as (1) dental education (videos about advantages and disadvantages of using rubber dams were played in the waiting room, operating procedures were shown as well). So that children and their parents could learn about rubber dams when waiting for medical treatment. This would deepen their knowledge on dental treatment and eliminate fear; [2] using children's language through the whole treatment [17]. To improve their comprehension and cooperation, nurses or dentists try to use some right age words to explain those steps, such as the word “umbrella or raincoat,” instead of “dam,” or “give tooth a shower” instead of “drill the tooth” [18]; [3] normalizing the practice: concentrated on learning the indications, contraindications, and standard operating methods for the rubber dams and conducted model exercises before clinical operation to enhance operating confidence; [4] experience sharing; and [5] local anesthesia. Many Chinese were contradicted to the anesthesia. In order to provide a pain-free comfortable treatment, guardian should sign the treatment informed consent and perform topical anesthesia or STA (single tooth anesthesia), so that the operation could be done thoroughly. When local anesthesia was rejected, topical anesthesia was also provided, by which discomfort could be relieved. Besides, some more new methods may be tried in future works [19].

Juntgen et al. [17] found that factors that hinder the application of new treatment methods in children's oral clinic include legality, parents' acceptance of changes, and limited resources. Through quality control circle activities, training of medical staff has been strengthened and popular dental education of children and parents has been enhanced. Besides, communication between medical staff and children and parents during diagnosis has strengthened, parents' acceptances of rubber dam application have been improved, and consumption of rubber dam has been effectively increased in root canal treatment of chronic pulpitis of deciduous teeth. Treating children usually involves a one-to-two relationship between doctors, children, and parents, that is, the pediatric dentistry treatment triangle [20]. After carrying out quality control circle activities, staff, parents, and children communicate more in details. And more communication makes the parents feel cherished, which may shorten the distance between medical staff and children and parents, may enhance mutual trust, and may improve children's obedience and the degree of satisfaction [21]. Children and parents in routine practice play a positive role in promotion of new technology project [22].

The article "Application of Quality Control Circle in Promoting the Use of Rubber Dams in the Root Canal Treatment of Primary Teeth" was retracted in 2024. Reasons: suspected computer-generated content; unreliable results or conclusions; concerns about the data; concerns about the results or conclusions.

Our department has achieved the target value through quality control circle activity, but there is still a gap between the usage of rubber dam in root canal treatment of deciduous teeth and that of permanent teeth. Compared with the 100% incidence rate of permanent root canal treatment, the incidence rate of pulpitis root canal treatment was only 67.35% (the specific data were not shown). This is mainly due to the treatment of young children with low degree of cooperation. When the defect of the child's teeth is too large (two walls are subgingival), or the child's head movement was too big, it is unable to spend a long time in the treatment of the child's teeth to pile up the tooth wall, which leads some doctors to give up the use of the rubber dam of the baby teeth. In order to promote the standardization of the entire activity results in production and normalized quality management, several ways have been tried to improve the rubber dam consumption. Different ring set have been used to fit special shape tooth, and in the second phase of circle activity, different brands of subgingival clamps or the small clips have been tried. The QCC group published monthly statistics, continued to carry out relevant training activities such as skills contest regularly, and summarized the work and the quarterly results into the department medical treatment appraisal system.

Children's personality, parents' appropriate preparation for the clinic, and excellent communication skills of medical staff are several key factors for the success of oral therapy [16]. For children who failed to accept the rubber dam after the first root canal treatment, parents should be instructed to provide effective comfort and communication to the children at home, and try to convey the information to the children and their parents through behavior management in the next visit [18], so as to improve the use of rubber dam of milk teeth. Besides, through the Houpt score evaluation system, it has been shown the children in treatment became more cooperative; in order to eliminate the possibility that children and parents who are willing to accept RD have a character of more cooperative and willingness to obey, in the further research, more questionnaires on parents and patients should be taken.

The article "Application of Quality Control Circle in Promoting the Use of Rubber Dams in the Root Canal Treatment of Primary Teeth" was retracted in 2024. Reasons: suspected computer-generated content; unreliable results or conclusions; concerns about the data; concerns about the results or conclusions.

Organizing and carrying out quality control circle activity not only improves work efficiency and causes economic benefits but also reduces medical risks and the working pressure of medical staff. As a way to improve the quality of clinical treatment, the effect of quality control circle activity is satisfactory. Through this quality control circle activity, the ability of medical staff in our department in finding, analyzing, and improving problems was enhanced. Through discussion, preparation, and implementation of corresponding countermeasures, the usage of rubber dam in root canal treatment of chronic pulpitis of deciduous teeth was greatly improved. The scientific research awareness and ability of the circle members have also been improved in the process of carrying out this quality control circle activity, which provides certain practical basis and experience guidance for the next quality control circle activities of our department.

## Figures and Tables

**Table 1:** Houpt's behavioral rating scale for rubber dam treatment.

Score	Description
1	Aborted, no treatment rendered
2	Poor treatment interrupted, only partial treatment completed
3	Fair treatment interrupted, but eventually all completed
4	Few treatment interrupted, but eventually all completed
5	Very good, some limited crying or movement (e.g., during anesthesia or mouth prop insertion)
6	Excellent, treatment completed

**Table 2:** Comparison of Houpt's score and clinical operation time between the two groups.

	Houpt's score (points)	Chairside operation time (min)
Experimental group	5.80 ± 0.52	13.20 ± 1.81
Control group	5.05 ± 1.01	18.58 ± 2.27

$P<0.01\;\left(\bar{\chi }\pm s\right)$.

**Table 3:** The comparison of intraoperative and postoperative complications between two groups.

	Experimental group (%)	Control group (%)
Intraoperative discomfort	10.00	0
Gingival bleeding caused by clamp	30.00	0
Mucosal bleeding caused by saliva suction	0	35.00
Provoke or vomiting	0	55.00
Postoperative discomfort	5.00	5.00

*P* < 0.01.

## Data Availability

The data used to support the findings of this study are available from the corresponding author upon request.
